# Novel Design and Optimization of Porous Titanium Structure for Mandibular Reconstruction

**DOI:** 10.1155/2022/8686670

**Published:** 2022-06-24

**Authors:** Renshun Liu, Yuxiong Su, Weifa Yang, Xiaobing Dang, Chunyu Zhang, Ruxu Du, Yong Zhong

**Affiliations:** ^1^Shien-Ming Wu School of Intelligent Engineering, South China University of Technology, Guangzhou 511400, China; ^2^Oral and Maxillofacial Surgery, The University of Hong Kong, Prince Philip Dental Hospital, Hong Kong SAR 999077, China; ^3^Guangzhou Janus Biotechnology Co., Ltd, Guangzhou 511400, China

## Abstract

A porous material is considered to be a potential material that can be used to repair bone defects. However, the methods of designing of a highly porous structure within the allowable stress range remain to be researched. Therefore, this study was aimed at presenting a method for generating a three-dimensional tetrahedral porous structure characterized by low peak stress and high porosity for the reconstruction of mandibular defects. Firstly, the initial tetrahedral porous structure was fabricated with the strut diameters set to 0.4 mm and a mean cell size of 2.4 mm in the design model space. Following this, the simulation analysis was carried out. Further, a homogenization algorithm was used for homogenizing the stress distribution, increasing porosity, and controlling peak stress of the porous structure by adjusting the strut diameters. The results showed that compared with the initial porous structure, the position of the large stress regions remained unchanged, and the peak stress fluctuated slightly in the mandible and fixation system with the optimized porous structure under two occlusions. The optimized porous structure had a higher porosity and more uniform stress distribution, and the maximum stress was lower than the target stress value. The design and optimization technique of the porous structure presented in this paper can be used to control peak stress, improve porosity, and fabricate a lightweight scaffold, which provides a potential solution for mandibular reconstruction.

## 1. Introduction

Treatment of large segmental bone defects in the mandible caused by trauma, benign or malignant tumor, remains a challenge for surgeons to date [1]. A microvascular-free fibular graft is considered to be the contemporary gold standard for the treatment of mandibular defects and has been widely used [2]. However, the shape and size of autogenous bone grafts differ significantly from that of mandibular defects, resulting in asymmetry of the postoperative facial contour and poor cosmetic effect on the patient [3, 4]. Complications associated with the donor site, such as a decrease in walking endurance and strenuous exercise, are also seen [5, 6].

Tissue engineering provides a solution for bone defects [7]. This new approach combines the advantages of both autografts and allografts and eliminates the problems of donor scarcity. Many studies were conducted on bone replacement materials due to limitations regarding biocompatibility, mechanical properties, and other factors. Metal materials (titanium alloy, cobalt-chromium alloy, 316L stainless, etc.) have become the most commonly used orthopedic materials. Ti6Al4V is still considered the optimal material for the production of orthopedic implants due to its excellent combination of corrosion resistance, biocompatibility, and mechanical properties [8, 9]. Moreover, the porous Ti6Al4V scaffolds with a wide range of morphological and mechanical properties can be made using additive manufacturing technology, which solves the difficulty in the preparation of mandibular prostheses [10, 11].

Compared to the natural bone, a solid titanium implant shows a stronger stiffness and elastic modulus, which induces a stress shielding effect on its surrounding bone that leads to an implant failure [12]. Implant porosity affects the displacement, stresses, and strain intensity of surrounding bone, and the selection of an appropriate implant according to the type of bone is conducive to improving safety [13]. Ideally, implants must be highly porous to decrease the stress shielding and allow the ingrowth of the new bone. In addition, a high porosity implant possesses strong permeability, which facilitates the easy diffusion of nutrients and the delivery of sufficient cellular mass for tissue repair [14, 15]. However, a high-porosity scaffold usually lacks mechanical strength and is prone to fatigue damage. Fatigue wear and fractures have been reported as the main problems during implant failure, and it remains difficult to design porous structures with high porosity within the allowable stress range [15–17]. Excellent design is a key factor in success. Otherwise, a longer healing time would lead to implant failure.

We reviewed articles on the design and optimization of mandibular scaffolds up to June 2021. Based on the design method and characteristics, the current approaches were divided into three categories. In type 1, the porous scaffolds were obtained by the Boolean operation between the uniform porous structure and the design model [18]. Free-ends and stepped surfaces are produced because the nodes of the periodic lattice structure show difficulty fitting the surface of the design model, resulting in a few risks during clinical use. Xiao et al. [19] designed a surface wrapping layer to apply on the surface of the porous structure to eliminate the free end; however, the semiclosed space is not conducive to the exchange of body fluids. In type 2, the mechanical properties of the scaffold could be improved by optimizing the plate configuration or combining topology optimization technology. The topological optimization design of the fixed structures of the porous mandibular scaffold was reported by Peng et al. [20], and the maximum stress of the optimized scaffold had decreased to 280.5 MPa. Cheng et al. [21] designed a customized support structure along the stress transfer path within the mandibular scaffold. The results indicated that the peak stress and weight of the optimized scaffold were reduced compared with that of the initial scaffold. Ferguson et al. [22] combined plate design with multiobjective optimization to determine the optimal height and angle to place a titanium fixation plate on a reconstructed mandible to enhance tissue ingrowth and structural mechanical properties. An ideal scaffold has high porosity and uniform stress that stimulates bone growth rather than merely reducing the peak stress. In type 3, novel design or optimization methods are used to homogenize the stress distribution of the scaffold. Luo et al. [23] reported a method of extracting mesh lines for designing a tetrahedral structure scaffold, which adopts the principle of stress homogenization techniques for optimization. The maximum stress of the optimized scaffold decreased, and the porosity increased in comparison to that of the initial scaffold. Although the peak stress decreases after optimization, it does not converge within the target stress. Gao et al. [24] proposed a 3D titanium scaffold design and optimization method, in which the strut diameters were optimized according to the azimuthal gradient through the general biomechanical analysis, the maximum stress of the optimized scaffold was reduced, and the stress distribution was more uniform. However, the maximum stress of the optimized scaffold was still high, and there was no analysis of porosity. To our knowledge, there is no excellent design and optimization method for a scaffold with smooth surfaces, controllable peak stress, and high porosity.

In light of previous studies [21, 23], a finite element method was proposed in this paper to design and optimize the tetrahedral porous structure for the repair of mandibular defects. The strut diameters of the porous structure were optimized as per the numerical simulation results. That is, high-stress struts are of large diameters, and low-stress struts are of small diameters to reduce material wastage as much as possible while maintaining their mechanical performance. The results showed that the maximum stress of the optimized porous structure was lower than the target stress value, and the porosity increased greatly, achieving the design goals. Furthermore, the controllable peak stress and high porosity structure design algorithm proposed in this paper is suitable not only for mandibular prosthesis but also provides a reference for the lightweight design of the other scaffolds.

## 2. Materials and Methods

### 2.1. Reverse Modeling and Implant Components

The preparation of the structural design for mandibular defects is shown in Figure 1. Data of a head CT scan was taken from a patient having oral squamous cell carcinoma as an example. Ethical approval and informed consent have been obtained for using the imaging data of the patient. The image contours of the maxilla and mandible were extracted using the Mimics 20.0 (Materialise, Belgien) to obtain the models of the triangular faces; then, the mandibular coordinates were registered according to the facial feature points. The defect mandibular model was repaired using the Geomagic Studio 2012 software (Geomagic, USA). To simplify the mandibular model, the dentition triangular slices were removed, and the cavities were sutured. Smooth the surface of the model and remove prominent features. Then, manually check and repair the cracks, reversals, and interference problems of the triangular slices to ensure the correctness of the mandibular model. After a series of reverse modeling procedures, the original triangular slice model of the mandible in the STL format was transformed into an IGES format.

The mandible resection planes were determined based on the tumor location by an experienced surgeon to obtain a design model (Figure 1). The plates were generated by trimming the entity, which was equidistant by 2 mm from the surface of the mandible, and the plate width was 8 mm. To reduce the effect of stress shielding, the plate was divided into two parts to facilitate stress transfer through the design model and connected to the surface of design model to form the scaffold. Six screws with a radius of 1.5 mm were used to fix the plates in the residual mandible, and the screws were all designed as cylinders to simplify the modeling process.

The detailed design assembly of the mandibular framework consisting of the residual mandible, design model, plates, and screws is illustrated in Figure 2(a). Classify and number plates and screws according to their position. The tetrahedral element was used to design the porous structure in the design model, and the size of the porous structure is shown in Figure 2(b).

### 2.2. Design of Porous Structure

The porous structure was performed by using the design model to achieve an anatomically correct contour. A three-dimensional tetrahedral structure was applied to the open porous structure, and the cell size and the strut diameter were selected as the design parameters. The initial mean cell size was chosen to be 2.4 mm. It has been previously reported that during selective laser melting fabrication process, the thickness of the minimum accuracy was approximately 10 *μ*m [25]. To guarantee the quality and connectivity of the porous structure, the lower and upper strut diameters were set to 0.3 mm and 0.6 mm (0.05 mm interval), respectively. The diameter of the strut of the initial porous structure was set at 0.4 mm.

The porous structure was designed using the Ansys 15.0 software (Dassult, USA) (Figure 3). Based on the initial parameters, the design model was decomposed into an approximately uniform tetrahedral mesh with an edge length of 2.4 mm. The node coordinates of the tetrahedral mesh and the connection relationship between each node were recorded to establish the model line structure by programming. Each connection line was replaced with a cylinder cross-section strut with a 0.4 mm diameter for the beam element, and the initial porous structure was obtained.

### 2.3. Biomechanical Evaluation of Porous Structures

All the materials were considered to be isotropic, linear elastic, and homogeneous for simplifying the finite element analysis. The porous structure was prepared by selective laser melting with the titanium alloy (Ti6Al4V), and the elastic modulus and the Poisson's ratio of material are 110 GPa and 0.3, respectively [26]. The remaining mandible was cortical bone with an elastic modulus of 15 GPa and a Poisson's ratio of 0.3 [27].

The plates were integrated with the porous structure to form the scaffold, and the contacts were made using the multipoint constraint algorithm. The reconstructed mandible was at a later stage, and the porous structure was fixed to the residual mandible. The cortical bone, plates, and screw were meshed with the tetrahedral element. To ensure the accuracy of the results, the mesh was refined in the regions having large feature mutations. The mesh sensitivity analysis results showed that the numerical simulation could converge precisely with the number of elements was 123268 in this study.

Finite element analysis was performed on a reconstructed model to evaluate the mechanical properties of the porous structure under physiological loading conditions (Figure 4). Two types of static loading states, incisal clenching (INC), and the left unilateral molar clenching (LMOL) were simulated. All fixes limited the degrees of freedom of the corresponding nodes, and all muscle forces were applied equally to the corresponding nodes on the mandibular surface. The values and directions of the normal muscle forces were obtained from relevant research [28, 29].

### 2.4. Optimization of the Porous Structure in Physiological Loads

After establishing the finite element model, the porous structure was optimized according to von Mises stress under the physiological loads. An optimization algorithm was proposed in this study to make the porous structure possess large porosity within the target stress range.

Within the porous structure, the struts meet the minimum weight requirements of the target stress range. The outer contour of the porous structure and the tetrahedral elements of the model remain unchanged, and the strut diameter is introduced as the design variable. The optimal design scheme was to achieve an expected goal among the feasible schemes to meet the requirements. The optimization process could be defined as follows:

(1) $$\begin{array}{c} \text{Find }D=\left[D_{1},D_{2},\cdots ,D_{n}\right],\\ \text{Min }W=\rho \overset{n}{\underset{i=1}{\sum }}\left(l_{i}A_{i}\right)=\frac{\pi \rho }{4}\overset{n}{\underset{i=1}{\sum }}\left(l_{i}D_{i}^{2}\right),\\ \sigma_{\max}=\text{Max}\left\{\sigma_{i}\right\}<\left[\sigma \right],i=1,2,\cdots ,n,\\ \text{S}.\text{t}.D_{i}\in \left\{0.3,0.35,\cdots ,0.6\right\}\text{mm},i=1,2,\cdots ,n, \end{array}$$

where *n* is the total number of struts in the porous structure. *W* is the weight of the porous structure, *ρ* is the density of the Ti6Al4V material, and the *l*_*i*_, *A*_*i*_, and *D*_*i*_ represent the length, cross-sectional area, and the diameter of the *i*th strut, respectively. *σ*_max_ denotes the peak stress of the porous structure, *σ*_*i*_ is the maximum stress of the *i*th strut, and [*σ*] represents the target stress of the porous structure. The strut diameters are between 0.3 mm and 0.6 mm (0.05 mm interval).

The optimization algorithm and the design process could be divided into several steps, and the pseudocode for the entire process is provided by the algorithm shown in Algorithm 1.

*k* is the number of iterations represented in Algorithm 1. *D*^(0)^ denotes the initial design, and its superscript represents the iteration number, and *D*_*i*_^(0)^ is the initial diameter of the *i*th strut, with *n* in total. The initial strut diameters were set to 0.4 mm (model A). *λ*^(*k*)^ is the iteration coefficient of the *k*th iteration. “SOLVE” stands for numerically solved finite element model. *σ*_*i*_^(*k*)^ is the peak stress value of the *i*th member in the *k*th iteration, and *σ*_*im*_^(*k*)^ is the maximum stress value of the *i*th strut during the *m*th loading in the *k*th iteration. *m* equals 1 is the incisal clenching, and *m* equals 2 is the left unilateral molar clenching, and *σ*^(*k*)^ is the peak stress at the *k*th iteration of the porous structure.

The optimization is aimed at realizing the homogeneous stress distribution of the porous structure within the target stress value, removing unnecessary materials, and increasing porosity. The maximum stress in the defect mandible was approximately 17 MPa under masticatory loads, and the elastic modulus of Ti6Al4V was about seven times that of the cortical bone. To produce the same stimulus for the peak strain, 120 MPa (model B) was considered as the target stress value. In addition, 100 MPa (model C) and 80 MPa (model D) were used as the target stresses for optimizing the porous structure for comparison. As a result, optimal porous structures were achieved.

The porosity of the porous structure was calculated using the following formula:

(2) $$\begin{array}{c} P=\left(\frac{V_{0}}{V_{S}}\right)\times 100\%=\left(1-\frac{V_{k}}{V_{S}}\right)\times 100\%, \end{array}$$

where *V*_0_ is the volume of the pores, *V*_*s*_ is the overall volume of the design model (7160.13 mm^3^), and the *V*_*k*_ is the volume of the entities. The volumes were measured automatically by the software.

## 3. Results

### 3.1. Mechanical Properties of Mandible and Fixation System

To obtain detail information about the influence of porous structure on mandible and fixation system, the results of the finite element analysis under two occlusal situations are shown in Figure 5. The distribution of the large stress areas of mandible and the fixation system was similar before and after the optimization of porous structure.  Figure 5(a) shows the stress distribution of each mandible and fixation system under INC occlusion. The high stress of the mandible was mainly distributed at both condylar necks and near the chin screw 3.  Figure 5(b) shows the stress distribution of the mandible and fixation under LMOL occlusion, and the high stress of the mandible was mainly distributed in right condylar neck. Peak stress of fixation occurred in chin screw 3 regardless of occlusal situations.  Figure 5(c) shows slight fluctuations in peak stress values of the mandible and fixation system under two occlusions before and after porous structure optimization.

### 3.2. Geometric Properties of Porous Structures

Figure 6 shows the geometric features of the porous structures. The outline of the porous structures was consistent with the design model, and the surface of the porous structure avoided stepped structures and free ends because the frame was not designed using Boolean subtraction, which represented a significant improvement with the design approach. The strut diameters of the porous structure are represented by seven colors, with warmer colors indicating larger diameters and colder colors signifying smaller diameters. In model A, the entire porous structure presented a relatively uniform mesh with all diameters of the struts being 0.4 mm with a porosity of 66.83%. Although the initial design parameters were the same, more and more struts showed large diameters with a decrease in the target stress value. The main reason is that when the target stress value is lower, a larger strut diameter is required to reduce the stress magnitude while decreasing porosity.  Figure 7 shows the distribution of strut diameter of the four porous structures. As the target stress decreased, the diameter increased for many more struts. However, most of the struts remain with the minimum diameter (0.3 mm). The porosity and minimum diameter strut ratio of the optimized structures were different: 80.31% and 92.1% for model B, 79.15% and 86.28% for model C, and 73.23% and 64.13% for model D, respectively.

120 MPa was considered to be a suitable target stress value for optimization, which stimulates the strain of the porous structure close to the natural mandible. The maximum strut diameter of the optimized porous structure (model B) was 0.55 mm. Compared to the initial porous structure, the number of strut diameter decreasing, constant, and increasing ratios were 96.07%, 2.24%, and 1.68%, respectively. The diameter was reduced for most of the struts, which was why the porosity of the optimized porous structure was greatly improved.

### 3.3. Mechanical Properties of Porous Structures

The biomechanical behaviors of the porous structures were compared under two separate occlusion conditions, and the after-effects of optimization were evaluated.  Table 1 shows the porosity and peak stress of the four porous structures. The peak stress within the initial porous structure was 91.69 MPa and 129.78 MPa under INC and LMOL loading, respectively. The maximum stress under LMOL loading was greater than that under INC loading in all porous structures. The peak stress of each of the optimized porous structures under INC and LMOL loading was lower than their corresponding target stress, and the porosity was greatly improved, so the plan was realized. The peak stress of model B was the highest among the three optimized porous structures. Its maximum strain (1074 *με*) in the numerical simulation was close to the mandibular defect. According to the theory of “the Mechanostat of the bone Biomechanics,” the stiffness of the porous structure adjacent to the surrounding bone could reduce the stress shielding, and the appropriate strain stimulated the growth of the bone tissue into the porous structure to maintain the dynamic balance. Furthermore, the peak stress of the porous structure was much less compared to the fatigue failure limit of Ti6Al4V, and none of the porous structures exhibited any risk of failure due to plastic deformation.

Figure 8 shows the stress distribution of model A and model B. They had a similar stress distribution under the same load, the peak stress was located in the upper part of the porous structure near the mandibular ramus during LMOL loading, and the high-stress struts were mainly concentrated on the surface of porous structure. According to the distribution of diameter (Figure 6) and von Mises stress (Figure 8) of the strut in model B, the stress magnitude distribution regions were consistent with the size of strut diameter, mainly due to the larger strut diameters were used for reducing the stress magnitudes in high-stress areas, while the smaller strut diameters were used for improving the porosity in low-stress areas. This improved the carrying capacity of the porous structure, avoided material waste, and resulted in uniform stress distribution.

The histogram of stress distribution for each strut in model A and model B under two mastication loads is shown in Figure 9. For model A, at least 75.62% of the struts were subjected to lower stress (less than 20 MPa), and model B decreased to 64.10%. The stress distribution of model B was more uniform under both INC and LMOL loading, and fewer struts were in a lower stress level.

### 3.4. Optimization Process

Figure 10 presents the variation in the peak stress value and the porosity during the optimization process when the target stress value was 120 MPa. After the first iteration, the peak stress and the porosity increased rapidly. As the iteration continued, peak stress and porosity of the porous structure decreased until the maximum stress was less than 120 MPa during the eighth iteration, and the iteration was stopped. Finally, the optimized porous structure showed an 8.98% reduction in peak stress and a 13.48% increase in porosity when compared to the initial porous structure. The results indicate that the optimized porous structure showed a better performance.

### 3.5. Additive Manufacturing of Porous Structures and Optimized Scaffold

The optimized scaffold, initial, and optimized porous structures were manufactured using the Ti6Al4V by selective laser melting (DiMetal-100, Laseradd, Guangzhou, China). The mass of the initial and optimized porous structures is 11.48 g and 8.17 g, which were measured by a high precision electronic balance. As shown in Figure 11, the optimized scaffold consists of the optimized porous structure and the plates, the struts were fully printed, and the connection was intact and highly interconnected, indicating that the sizes of the porous structures selected in this study were reasonable and manufacturable.

## 4. Discussion

An excellent scaffold for rebuilding the large segmental defects of the mandible needs to restore the facial profile and bear the repeated forces generated during the process of mastication. It is generally agreed that scaffolds must have the following characteristics [30, 31]: (i) perfect biocompatibility; (ii) mechanical properties that match the defected bone; and (iii) a highly porous and interconnected structure to allow cell migration, proliferation, differentiation, and nutrient-waste exchange.

The complex shape of the mandible makes it difficult for autologous bone transplantation to match the defect of the mandible. With the development of computer-aided design/manufacturing technologies, porous scaffolds provide a new option for mandibular reconstruction. Mandibular models could be obtained by CT images of the patients. Mandibular defect is separated and repaired to obtain the external contour of the design model. In previous studies, Boolean operations were used for generating the porous structure between the periodic lattice structure and the design model that led to a large number of free ends, presenting a step-like character. Furthermore, the global strut size of the porous structure is generally set to resist peak stress, resulting in a smaller porosity.

In this study, a tetrahedral structure was applied to design a porous structure. Tetrahedral trusses present some advantages. For example, most complex models can be meshed using tetrahedral structures to obtain struts that are consistent with the outer contours of the design models, avoiding the Boolean operations that produce the free ends on the surface of the porous structure. More importantly, the tetrahedral porous structure has good stability and is interconnected. Study has shown that the pore sizes varying between 200 *μ*m and 1200 *μ*m were optimum for tissue generation [32]. The occlusion rate of the Ti6Al4V implant of the pore size ranging from 450 to 1200 *μ*m was tested by Warnke et al. [33], the results showed that there was a decreasing proportion of occlusion with increasing pore sizes, and no occlusion was observed in the samples having large pore sizes (900–1200 *μ*m). Pore sizes were derived from the diameter of a circle inscribed using pore shapes, and a cell size of 2.4 mm is an excellent value in our research to design a porous structure with a large pore size that does not exceed the upper limit. Considering the accuracy of the selective laser melting technology, the lower limit of the strut diameter is set at 0.3 mm to ensure the quality of the porous structure forming. The upper limit of the diameter of the strut is determined by the load of the strut. When all the strut diameters are 0.6 mm, the maximum stress of the porous structure was about 63 MPa, which was lower than the target stress. Thus, the strut diameter setting meets the design requirements. A lower upper limit of the strut diameter could reduce the convergence speed and would even fail to obtain the optimal solution, while a higher upper limit of the strut diameter would cause partial pores to shrink or even close, which should be avoided.

Numerical simulation was used to evaluate the results of the porous structures under the two mastication conditions in this study. Changes in muscle strength before and after mandibular reconstruction remain unclear, and there are only a few reports regarding this aspect. We consider an ideal situation where muscle forces are attached to the surface of the bone and are aligned in size and direction with healthy mandibular muscle forces. The accuracy of the finite element model was improved by refining the mesh of prominent feature areas, and the validity of the model was confirmed by analyzing with different number of elements. The porosity of the initial porous structure was 66.83%, which is less than the average porosity of the components for orthopedic use (75–85%) [34]. The maximum stress was 129.78 MPa. The strain was slightly higher than the peak strain of mandibular defect. Most of the struts were at low-stress levels and a few at high-stress levels, indicating that most of the strut materials were insufficiently utilized and a few were overutilized. The initial strut diameter of the porous structure could be adjusted using the design range to realize the optimization of the porous structure.

The homogenization optimization algorithm is used to adjust the size of the porous structure and reduce the mass, and it has been researched and used in structural mechanics. Luo et al. [23] used a similar method to optimize porous scaffolds and achieved remarkable results, improving the utilization rate of scaffold materials. To obtain a high-porosity structure and to make the peak stress of the porous structure lower than that of the target stress value, an algorithm was proposed in this paper to adjust the strut diameter during iteration until the peak stress was lower than the target stress. During the same occlusal loading, the large stress distribution in the mandible and fixation system of the optimized scaffold was consistent with that of the initial scaffold, concentrated mainly at the condylar neck and chin screw 3, and the fluctuation of the maximum stresses was also limited (Figure 5). The rule of variation of the peak stress and the porosity of the porous structure during the iteration process is shown in Figure 10. After the first iteration, the porosity of the structure had improved greatly, but the peak stress of the porous structure under the mastication loads was still higher than the target stress; repeated adjustments of the strut diameter were still needed and had to be iterated to find a solution to reach the initial optimization goals. The optimized porous structure was obtained after 8 iterations, the porosity of the optimized structure was improved by 80.31%, and the peak stress decreased to 118.12 MPa. 92.10% of the struts were within the minimum allowable diameter (0.3 mm), and at least 64.10% of the struts were at the low-stress level (less than 20 MPa). The stress distribution of the porous structure was similar even before and after optimization, and the stress distribution of the optimized porous structure was not very homogeneous. This could be primarily attributed to the limitation of the strut diameter range. Struts having low-stress levels could not be changed to smaller diameters and vice versa. It was believed that with the development of additive manufacturing technology, a smaller strut diameter would have alleviated this problem. Although the optimization algorithm did not obtain an optimal global solution, the optimized structure showed that the porosity was higher, the peak stress was lower than the target stress, and the stress distribution was more uniform in the comparison between the initial structure and the optimized structure, which proved that the proposed optimization method was effective and feasible.

The target stresses of the other two control groups were 100 MPa and 80 MPa, respectively. Peak stresses were lower than their corresponding target stress. As the target stress decreases, the partial diameter of the strut increased, and the porosity decreased. However, compared with the initial porous structure, the porosity of all optimized structures increased (Table 1). In theory, too little stress would not produce enough strain to stimulate bone growth, resulting in stress shielding, while appropriate strain leads to osteogenesis and maintenance. The target stress of 120 MPa is far lesser than the fatigue failure limit of Ti6Al4V (900 MPa), and the peak strain generated by the optimized porous structure is close to the mandibular defect during chewing. Finally, the target stress of 120 MPa was selected as the optimal porous structure.

In recent years, magnesium has been considered a potential bone replacement material due to its excellent biocompatibility, biodegradability, and sufficient mechanical support [35]. However, the application of magnesium alloys is limited due to their difficulty in processing and gas generation during biodegradation [36]. With the development of research and processing technology, magnesium alloys may serve as a perfect alternative material for orthopedic implants [37, 38]. In any case, it takes decades for the transition of a new material to move from the laboratory to the clinic, and titanium remains the ideal alternative for bone material until a more enhanced version is put to use.

Regarding the limitation of this study, firstly, the mechanical model between dentition and the mandibular ramus is difficult to predict, and this study only considered the ideal condition in which the load applied to the dentition was applied to the surface of the mandible. Secondly, there are only a few reports on muscle force after mandibular reconstruction, and thus, it is unclear whether this has any effect on the force exerted by the muscles. We only consider the ideal case, and that there is no change in muscle strength before and after reconstruction. Thirdly, this study only considered the most commonly INC and LMOL loads; however, in some uncommon extreme occlusal loads, the instantaneous peak stress of the porous structure may exceed the target stress value. Fortunately, the target stress (120 MPa) of this research is far lower than the fatigue failure limit (900 MPa) of Ti6Al4V, which ensures the safe use of porous structure. Finally, this research assumed that the bone union was at a later stage. That is, the porous structure had adhered to the mandible. However, the combination of porous structure and mandible is dynamic, and more healing stages need to be considered to evaluate the mechanical properties of a porous structure.

## 5. Conclusion

In this work, an optimization algorithm for a tetrahedral porous structure having controllable peak stress and high porosity was proposed based on finite element design and simulation. A defected mandible is taken as an example, the porous structure was designed with a suitable pore shape and size, and the strut diameters were optimized under two different mastication loads. The numerical simulation results showed that the optimization of the porous structure had little effect on the stress distribution and maximum stress value of mandible and fixation system. The peak stress of the optimized porous structure was lower than the target stress value, and the porosity increased. The optimized porous structure with appropriate peak stress to prevent fatigue failure and higher porosity to increase permeability is a good choice for mandibular reconstruction. However, mandibular prosthesis design is a complex issue that has puzzled researchers for a long time, and thus, more supporting materials are still required. For example, mechanical tests and the corresponding animal experiments on mandible segmental defects are necessary procedures.

## Figures and Tables

**Figure 1:** Mandible preparation and implant design.

**Figure 2:** Implant components. (a) Partial view of the assembled implant attached to the mandibular framework. (b) Dimensions and minimum unit cell of the porous structure.

**Figure 3:** Tetrahedral porous structure formation process. (a) Design model. (b) Design model for tetrahedral meshing. (c) Extraction mesh lines. (d) Struts replace mesh lines to generate a porous structure.

**Figure 4:** Muscular forces (blue arrow) and constraints (triangle) applied in finite element simulation. Simulating the incisal clenching (INC) and left unilateral molar clenching (LMOL), respectively. SM: superficial masseter; DM: deep masseter; MP: medial pterygoid; AT: anterior temporalis; MT: middle temporalis; PT: posterior temporalis.

**Figure 5:** Von Mises stress distribution to the mandible and fixation under (a) INC loading and (b) LMOL loading and the (c) line chart of their peak stress.

**Figure 6:** Geometric features of the porous structures. The seven colors represent different strut diameters, ranging from 0.3 mm to 0.6 mm.

**Figure 7:** Strut diameter distribution of each porous structure.

**Figure 8:** Von Mises stress in model A and model B under INC and LMOL loading.

**Figure 9:** Stress distribution of model A and model B under INC and LMOL clenching.

**Figure 10:** Variation of peak stress and porosity during the iteration process when the target stress was 120 MPa.

**Figure 11:** Details of the printing of the optimized porous scaffold.

**Algorithm 1:** Optimization algorithm of strut diameter (0.05 mm interval).

**Table 1:** The performance parameters of four porous structures, including the porosity and the peak stress under two different clenching loadings.

	No.	Target stress (MPa)	Porosity (%)	Peak von Mises stress (MPa)	
				INC	LMOL
Model A	1	-	66.83	91.69	129.78
Model B	2	120	80.31	87.57	118.12
Model C	3	100	79.15	76.08	99.76
Model D	4	80	73.23	58.52	79.87

## Data Availability

The simulation data during the current study are available from the corresponding author on reasonable request.
